The article "The data dimensionality reduction and bad data detection in the process of smart grid reconstruction through machine learning" was retracted in 2025. Reasons: unreliable results or conclusions; concerns about the results or conclusions; concerns about the peer review.

# The data dimensionality reduction and bad data detection in the process of smart grid reconstruction through machine learning

**DOI:** 10.1371/journal.pone.0237994

**Published:** 2020-10-07

**Authors:** Bo Yu, Zheng Wang, Shangke Liu, Xiaomin Liu, Ruixin Gou

**Affiliations:** State Grid Ningxia Electric Power, Eco-Tech Research Institute, Yinchuan, China; University College London, UNITED KINGDOM

## Abstract

To detect false data injection attacks (FDIAs) in power grid reconstruction and solve the problem of high data dimension and bad abnormal data processing in the power system, thereby achieving safe and stable operation of the power grid system, this study introduces machine learning methods to explore the detection of FDIAs. First, through the utilization of the standard IEEE node system and the simulation of FDIAs under the condition of non-complete topology information, the construction of the attack data set is completed, and the MatPower tool is applied to simulate and analyze the data set. Second, based on the isolated Forest (iForest) abnormal score data processing algorithm combined with the Local Linear Embedding (LLE) data dimensionality reduction method, an algorithm for data feature extraction is constructed. Finally, based on the combination of the Convolutional Neural Network (CNN) and the Gated Recurrent Unit (GRU) network, an algorithm model for FDIAs detection is constructed. The results show that in the IEEE14-bus node and IEEE118-bus node systems, the overall distribution of the state estimated before and after the attack vector injection is consistent with the initial value. In the iFores algorithm, the number of iTree and the number of samples affect the extraction of abnormal score data. When the number of iTree n is determined to be 100, and the corresponding number of samples w is determined to be 10, the algorithm has the best detection effect. The FDIAs detection algorithm model based on CNN-GRU shows good detection effects under high attack intensity, with an accuracy rate of more than 95%, and its performance is better than other traditional detection algorithms. In this study, the bad data detection model based on deep learning has an active role in the realization of the safe and stable operation of the smart grid.

## 1. Introduction

Since 2019, the development and promotion of the ubiquitous power Internet of Things have promoted the enhancement of the intelligent power system; thus, the consequences of information security accidents caused by network attacks also become more serious [1]. For example, due to network attacks, a power bureau suffered severe economic losses [2]. The Supervisory Control And Data Acquisition (SCADA) industrial control system, which is widely utilized in power systems, is extremely vulnerable to hacker attacks [3]. In addition, the Sichuan-Chongqing Power Grid of China was severely damaged due to the shutdown of the Sichuan Ertan Hydropower Plant caused by abnormal signals. The concept of False Data Injection Attacks (FDIAs) was proposed in 2009. Then, the traditional state estimation bad data detection was widely applied [4, 5]. FDIAs greatly affect the normal and stable operation of power systems. Therefore, how to accurately detect FDIAs based on the attack characteristics is the focus and difficulty of the power system research. The detection of FDIAs has been studied all over the world. Research has shown that the classification of power measurement values can complete the construction of attack vectors at the lowest cost [6]. The design of multiple state variables and power measurement attack vectors can make the detection of FDIAs more operable [7]. Much work has been done on the topology information of the power network. Some scholars found that even under the condition of incomplete network topology information, FDIAs can still achieve the construction of attack vectors [8]. With the help of some power measurement vectors, some scholars have applied the subspace method under the premise of not fully understanding the network topology to the construction of FDIAs attack vectors. Globally, due to power outages caused by attacks, the concept of power CPS and attack, and a collaborative plan for the prevention of FDIAs have been proposed [9]. A greedy algorithm for power measurement data has significantly improved the detection efficiency of FDIAs [10]. Based on the Kalman filtering, some scholars have completed the design of FDIAs detection methods [11]. In summary, based on FDIAs, a variety of new types of FDIAs have appeared one after another, and they can be attacked at a low cost. This poses a growing threat to the safe and stable operation of power systems. Some FDIAs are implemented by injecting attack vectors into the false data of power measurement; however, it is difficult to complete the attacks on state variables. Similar traditional detection methods are difficult to detect FDIAs with massive data.

The article "The data dimensionality reduction and bad data detection in the process of smart grid reconstruction through machine learning" was retracted in 2025. Reasons: unreliable results or conclusions; concerns about the results or conclusions; concerns about the peer review.

On this basis, this study innovatively introduces the isolated Forest (iForest) algorithm and Local Linear Embedding (LLE) method based on machine learning, and completes the feature extraction of FDIAs data. Then, based on Convolutional Neural Network (CNN) and Gated Recurrent Unit (GRU) network, an algorithm model for FDIAs detection is established. This study aims to expand the application of machine learning methods in power systems, thereby providing a reference for the FDIAs detection in bad data detection of power systems.

## 2. Literature review

### 2.1 Research on FDIAs worldwide

Scholars worldwide have discussed and studied FDIAs. Mohammadpourfard et al. (2017) used the actual load data provided by independent system operators in New York and tested them on the IEEE 14-node and IEEE 9-node systems, respectively; the results showed that the method had a positive role in improving the stability of the power grid [12]. Beg et al. (2017) proposed a framework for detecting possible FDIAs in the physical DC microgrid of the power electronic dense DC microgrid and transformed the detection problem into the identification of changes in a group of inferred candidate invariants [13]. Ganjkhani et al. (2019) proposed a new bad data detection processor for identifying FDIAs in power system state estimation. The results show that the data detection processor could accurately detect false data injected into the system [14]. Moslemi et al. (2018) used malicious data market participants to interfere with the operation of the electricity market by using pre-designed FDIAs, as well as false electricity transactions in the current market; the attack design was robust to market uncertainty [15]. Hossein and Taghi (2018) proposed three indicators for detecting FDIAs; these indicators were based on three factors: the performance of the traditional power system, the relationship between the angle and the voltage change in each bus, and the performance of the neighbor bus; after testing, it was found that the three indicators showed good results in the attack detection of the smart grid [16].

### 2.2 Research on FDIAs in China

In China, many scholars have also discussed and studied FDIAs. Wang et al. (2019) used the measured value in the phasor measurement unit as the object of attack and defense in the power system and adopted the load reduction caused by the line fault to quantify the consequences of the attack to achieve effective defense against FDIAs [17]. Chen et al. (2019) revealed the potential connection between data attacks and physical consequences in the smart grid and analyzed the ways in which attackers launched malicious data attacks; this attack mechanism integrated the construction of optimal data attacks and identification of key lines, which had greater security and probability of occurrence [18]. By replacing the traditional pre-calculated thresholds with adaptive thresholds, Wang et al. (2019) proposed a distributed isolation scheme for adjacent grid partitions of FDIAs and verified the effectiveness of the scheme [19]. Shang et al. (2019) proposed a formal model of multi-device FDIA in the air traffic control system for location verification; it was found that the model had low cost and strong concealment, and could obtain better time synchronization to bypass the current anomaly detection [20]. Zhang et al. (2018) discussed and analyzed the physical consequences of unobservable FDIAs designed by the internal information of the power system subnet, and established a multiple linear regression model to learn the relationship between the external network and the attack subnet from historical data; taking the IEEE 14-node and IEEE118-node systems as examples, the vulnerability of the attack model was illustrated [21].

The article "The data dimensionality reduction and bad data detection in the process of smart grid reconstruction through machine learning" was retracted in 2025. Reasons: unreliable results or conclusions; concerns about the results or conclusions; concerns about the peer review.

The above analysis can reveal that FDIAs had a great influence on the smart grid. Although there have been many research results in this field, there is little research work on applying artificial intelligence-based machine learning methods to them.

## 3. Methods and experiments

### 3.1 Construction of FDIAs data set

In the detection of bad data, the bad data detection mechanism based on state estimation and power flow calculation rely on the setting of the threshold to eliminate the bad measurement data value. However, no matter how small the threshold setting is, it still cannot avoid the attacker escaping the detection of bad data by constructing the injection vector [22]. Under the FDIAs based on complete topology information, if the data attacker has completely mastered the power grid topology, the construction of the attack vector is very easy to realize. However, in reality, only the core personnel of the control center can fully master the complete network topology of the power system; most attackers can only master the local network topology and local power system parameters. Existing studies have found that based on the conditions of incomplete network topology information, FDIAs can still be successfully constructed. In the process of attack detection, FDIAs under incomplete topology information is considered, which is more practical. Therefore, based on the condition of non-complete topological information, the sample data is finally obtained by constructing false injection attack vectors and combining power measurement data.

If the attack detection model can be successfully implemented, the training set and test set of normal and negative power measurements, as well as the training set and test set of the post-attack positive and negative power measurement, are the basis. This study uses a standard IEEE node to obtain the measurement data in a normal state. Then, the FDIAs under the condition of the incomplete topology information of the attacker is simulated to obtain positive and negative data samples before and after the attack. By generating standard IEEE14-bus node and IEEE118-bus node systems with the help of MatPower tools, the required measurement data are obtained, and 20,000 measurement data at the corresponding time are generated in each of the two node systems. Besides, the measurement data after the FDIAs attack are constructed; thus, in the course of training and experiments, the IEEE14 and IEEE118 node systems each contain 40,000 pieces of power measurement data, and the measurement data of different node systems include 30,000 training samples and 10,000 test samples, respectively. The injection vector of FDIAs is represented by a, the measurement matrix is represented by *H*, the corresponding attack vector is represented by *b*, and the corresponding measurement error is represented by *e*; then, after the attack is launched, the corresponding measurement value *z*_*b*_ is:

$$z_{b}=H\text{x}+b+e$$ (1)

The measurement value is decomposed into *d* sub-regions; then, the linear expression of the state estimation can be expressed as:

$$\left[\begin{array}{c} z_{b1}\\ z_{b2}\\ \vdots \\ z_{bd} \end{array}\right]=\left[\begin{array}{c} H_{1}\\ H_{2}\\ \vdots \\ H_{d} \end{array}\right]x+\left[\begin{array}{c} b_{1}\\ b_{2}\\ \vdots \\ b_{d} \end{array}\right]+\left[\begin{array}{c} e_{1}\\ e_{2}\\ \vdots \\ e_{d} \end{array}\right]$$ (2)

Where: *z*_*bi*_ represents the measurement data corresponding to the *i*-th sub-region in the measurement matrix *H*_*i*_ after being attacked, *b*_*i*_ represents the attack vector in the corresponding sub-region, and *e*_*i*_ represents the measurement in the corresponding sub-region error. At this time, the residuals of all regional state estimates are expressed as:

$$\text{r}=\sum_{i=1}^{d}r_{i}={\|z_{b}-H\overset{\wedge }{x_{b}}\|}_{2}^{2}$$ (3)

Where: *r*_*i*_ corresponds to the residual of the *i*-th area, $\overset{\wedge }{x_{b}}$ represents the state variable in the area. Then, the best attack vector is constructed so that the residual after being attacked is the smallest, the corresponding expression is:

$$\min\sum_{i=1}^{d}r_{i}+\lambda \|\beta \|$$ (4)

Where: λ represents the regularization parameter, β corresponds to the optimization amount; thus, under the condition of incomplete network topology information, the correspondence between *a* and *b* is:

$$\left[\begin{array}{c} \overset{\wedge }{b_{1}}\\ \overset{\wedge }{b_{2}}\\ \vdots \\ \overset{\wedge }{b_{d}} \end{array}\right]=\left[\begin{array}{c} \overset{\wedge }{H_{1}}\\ \overset{\wedge }{H_{2}}\\ \vdots \\ \overset{\wedge }{H_{d}} \end{array}\right]\times \left[\begin{array}{c} a_{1}\\ a_{2}\\ \vdots \\ a_{d} \end{array}\right]$$ (5)

To find the optimal solution of *a*, solving the following function can obtain the attack injection vector of FDIAs under the condition of non-complete network topology:

$$\min{\sum_{i=1}^{d}\|b_{i}-H_{i}a_{i}\|}_{2}^{2}+\lambda \|\theta \|$$ (6)

Where: θ represents the optimized variable, and the vector *a* is injected into the standard IEEE14-bus node and IEEE118-bus node systems. This vector can annotate the measurement data samples under attack and normal measurement data samples under the Python environment, and finally, generate training samples and test samples. It is expressed as data set *D*:

$$D=\left\{X,Y\right\}=\left[\left(x_{1},y_{1}\right),\left(x_{2},y_{2}\right),\cdots ,\left(x_{4000},y_{20000}\right)\right]$$ (7)

Where: *X* corresponds to the sample of the attack detection measurement data, and *Y* represents the label of the sample category.

The article "The data dimensionality reduction and bad data detection in the process of smart grid reconstruction through machine learning" was retracted in 2025. Reasons: unreliable results or conclusions; concerns about the results or conclusions; concerns about the peer review.

### 3.2 Data feature extraction based on iForest and LLE

The measurement data in the power system have the characteristics of high dimensionality and nonlinear structure [23]. They are difficult to be directly applied to the training and detection of the model. In the dimensionality reduction of high-dimensional data, machine learning is widely utilized. If only the dimensionality reduction processing is performed on the measurement data, it cannot ensure the pertinence of attack detection. Considering that the attack method of FDIAs is tampering with the measurement data, and the data after the attack is random, the data before and after the attack has data distribution or outliers. Therefore, in the data processing stage, this study uses the method of abnormal score extraction to quantify the outlier characteristics of the measured data. iForest is an integrated learning algorithm for anomaly detection. It can calculate anomaly score data without building a data model. At the same time, the algorithm has the characteristics of high calculation efficiency and high detection stability [24]. The algorithm consists of a large number of iTrees; the entire process is completed in the multiple sampling of the measurement data set, which is applicable to large-scale complex power measurement data. After being established, the iForest can output the abnormal score corresponding to each piece of power measurement data. The basic principle is that if the average traversal depth of power measurement data sample x in all iTrees is greater, the corresponding abnormal score will be smaller, and vice versa. Therefore, the quantitative equation for the anomaly score is defined as follows:

$$c\left(\mu \right)\{\begin{array}{cc} 2H\left(\mu -1\right)-\left(2\left(\mu -1\right)/n\right) & ,\mu >2\\ 1 & ,\mu =2\\ 0 & ,\mu <2 \end{array}$$ (8)

H(t)=ln(t)+ζ (9)

Where: ζ represents Euler’s constant, and the expression of the iForest anomaly score corresponding to each data sample *x* is:

$$iscore\left(x\right)=2^{\frac{-E\left[h\left(x\right)\right]}{c\left(\mu \right)}}$$ (10)

Where: *h*(*x*) represents the path length of *x*, and *Eh*(*x*) represents the average path length on all iTree.

The article "The data dimensionality reduction and bad data detection in the process of smart grid reconstruction through machine learning" was retracted in 2025. Reasons: unreliable results or conclusions; concerns about the results or conclusions; concerns about the peer review.

In the detection of FDIAs, when the abnormal score *iscore*(*x*) is used as an independent feature, the abnormal score power measurement data after feature extraction is still in a high-dimensional state; thus, further feature extraction is needed.

LLE is an unsupervised dimensionality reduction method for nonlinear structural data. The local reconstruction weight matrix is established by considering the data points in the locally linear structure [25], thereby considering the maintenance of the structure and the search for the low-dimensional mapping under the high-dimensional data. Due to the few parameter settings in the realization process, it is easy to realize; thus, it is consistent with the characteristics of the high-dimensional data of electric power. The completion of data dimensionality reduction includes the search for the distance between sample points and adjacent points in high-dimensional space, and the construction of local reconstruction weight matrix and the establishment of mapping from high-dimensional space to low-dimensional space. The calculation for the distance between the original high-dimensional data point *x*_*i*_ and the adjacent point is:

$$d_{ij}=\sqrt{\sum {\left(x_{ik}-x_{jk}\right)}^{2}}$$ (11)

Where: *k* represents the number of adjacent points. Based on the Lagrangian multiplier method, the construction of the local reconstruction weight matrix is:

$$\omega_{ij}=\frac{\sum_{m=1}^{k}{\left(Q^{i}\right)}_{jm}^{-1}}{\sum_{p=1}^{k}\sum_{q=1}^{k}{\left(Q^{i}\right)}_{pq}^{-1}}$$ (12)

Where: ω_*ij*_ represents the local weight matrix, and *Q*^*i*^ is the singular matrix. To realize the data mapping from the high-dimensional space to the low-dimensional space, the establishment of the objective function is:

$$\min P\left(Y\right)={\sum_{i=1}^{N}|y_{i}-\sum_{j=1}^{k}\omega_{ij}y_{ij}|}^{2}=\sum_{i=1}^{N}\sum_{j=1}^{N}M_{ij}y_{i}^{T}y_{j}$$ (13)

$$M={\left(I-W\right)}^{T}\left(I-W\right)$$ (14)

Where: *y*_*i*_ and *y*_*j*_ correspond to data points in low-dimensional space, *I* is the identity matrix, and *W* is the local reconstruction weight matrix.

On this basis, the advantages of iForest and LLE in anomaly detection and high-dimensional data reduction are combined, and a feature extraction method for iForest-LLE power measurement data for FDIAs detection is proposed. The implementation process of the iForest-LLE algorithm is shown in Fig 1. First, the anomaly score iscore(x) corresponding to each piece of data extracted by the feature is regarded as an independent feature, and then LLE is used to reduce the dimensionality of the data in the specified dimension r for high-dimensional data. The classification of features is comprehensively calculated, and the measurement data feature *P* for data attack detection is defined as:

$$P=\left[ID,iscore\left(x\right),f_{1},f_{2},\cdots ,f_{r}\right]$$ (15)

Where: *ID* corresponds to the number of the data sample, and [*f*_1_, *f*_2_, *L*, *f*_*r*_ ] is the new attribute corresponding to the power measurement data after *LLE* dimensionality reduction processing.

The article "The data dimensionality reduction and bad data detection in the process of smart grid reconstruction through machine learning" was retracted in 2025. Reasons: unreliable results or conclusions; concerns about the results or conclusions; concerns about the peer review.

**Fig 1:** iForest-LLE algorithm implementation.

### 3.3 Data attack detection model based on CNN

Machine learning uses computers to simulate human learning behaviors. It has the ability to classify and predict. It belongs to the field of artificial intelligence. It has been widely used in fields such as speech recognition, image processing, and data mining. Its implementation includes supervised and unsupervised learning, in which the prediction accuracy of supervised learning is the highest [26]. In addition, its tasks include classification and regression. Therefore, it is the most used. At the same time, the detection of FDIAs is essentially a typical classification task. In general, the selection of algorithms and the quality of training data are critical in predicting the effect. Most machine learning algorithms, including neural networks, decision trees, and support vector machines, can consider both classification and regression tasks, but the final effect is very different. In recent years, deep learning methods have been gradually applied to the detection of data integrity attacks. Due to the complex scenes and high noise characteristics of the power system network environment, the detection performance of traditional shallow machine learning algorithms will be affected and reduced when the amount of data is relatively large. Meanwhile, the deep learning algorithm can achieve the classification of a large number of extracted data features; therefore, the efficiency is higher, and it will be more reliable. On this basis, this study organically combines CNN and GRU and proposes a data integrity attack detection model based on the hybrid neural network.

The traditional CNN method is often used to extract image space features [27]. At the same time, the data integrity attack is closely related to the topology information of the power grid structure. Combining CNN and GRU can realize the synchronous feature extraction of the corresponding space and time for the attack sample. The implementation of the FDIAs attack detection model based on the CNN-GRU hybrid network constructed in this study is shown in Fig 2 below.

The article "The data dimensionality reduction and bad data detection in the process of smart grid reconstruction through machine learning" was retracted in 2025. Reasons: unreliable results or conclusions; concerns about the results or conclusions; concerns about the peer review.

**Fig 2:** Implementation of FDIAs attack detection model based on CNN-GRU hybrid network.

The detection model mainly includes a training phase and a detection phase, in which the training phase completes feature extraction based on the original data of the attack samples to obtain an appropriate data integrity attack signature database; the detection phase inputs the collected real-time data into the hybrid network and completes the classification of related data with the help of softmax classifier. The traditional CNN network is composed of a data input layer, a convolutional layer, a pooling layer, a fully connected layer, and a data output layer. In the design of the CNN-GRU hybrid network, 100 GRU structures are added before the fully connected layer of the traditional CNN network, thereby realizing the processing of the timing characteristics of the input data. A separate GRU is composed of an update gate and a reset gate. After the CNN-GRU hybrid network is trained, it can detect power data integrity attacks. First, the initial measurement data set {*z*_*t*_} is preprocessed. Then, the matrix *Z* is obtained by processing the measured value vector

$$Z=\left[\begin{array}{cccc} z_{1,1} & z_{1,2} & \cdots & z_{1,m}\\ z_{2,1} & \cdots & \cdots & z_{2,m}\\ \cdots & \cdots & \cdots & \cdots \\ z_{n,1} & z_{n,2} & \cdots & z_{n,m} \end{array}\right]$$ (16)

As the input of the hybrid network, the data are normalized, and the pre-processed input layer data are input into the convolutional layer; the result of the convolutional layer is input into the pooling layer. In addition, the data are divided into non-overlapping areas according to the size of the window. Afterward, the appropriate window size is selected according to the size of the data to perform the pooling operation, thereby achieving the dimensionality reduction of the feature. After repeating the previous steps many times, the final results are input into 100 GRU network structures; finally, the data are input into the fully connected layer through the update gate and reset gate. The classification is completed through the softmax classifier, and the final result is output. The realization of the corresponding detection process of the detection model is shown in Fig 3 below.

**Fig 3:** Implementation of the model checking process.

### 3.4 Selection of evaluation indicators

In this study, accuracy (Ac) is selected as the evaluation indicator for power data integrity detection. The meaning of Ac is the ratio between the number of all correctly judged samples and the overall number. The higher the Ac value is, the more effective the algorithm model is. Ac is defined as:

$$Ac=\frac{TN+TP}{TN+FN+TP+FP}$$ (17)

Where: TN represents the number of normal data identified as normal data, TP represents the number of problem data identified as problem data, FN represents the number of normal data identified as problem data, and FP represents the number of problem data identified as normal data.

The article "The data dimensionality reduction and bad data detection in the process of smart grid reconstruction through machine learning" was retracted in 2025. Reasons: unreliable results or conclusions; concerns about the results or conclusions; concerns about the peer review.

To verify the effectiveness of the detection model, the IEEE 14-bus node and IEEE 18-bus node system are selected as the test environments; in addition, the MatPower tool is chosen. Based on the selected evaluation index, the attack dataset, iForest-LLE data feature extraction, and data attack detection models are simulated and analyzed. In the analysis of the effect of the attack detection model, the traditional Deep Belief Network (DBN) algorithm is chosen for comparative analysis [28].

## 4. Results

### 4.1 Simulation analysis of attack data set

The MatPower tool is utilized to set the FDIAs vector a to 3 and perform injection attacks on the IEEE14-bus node and IEEE118-bus node systems, respectively. The corresponding state estimates of the node system before and after the attack are changed, as shown in Fig 4 below.

**Fig 4:** Changes in state estimates before and after a node system undergoing an attack.

As shown in the figure, after the IEEE14-bus node system is injected with the attack vector, the corresponding state estimate is shifted upward from the initial amount. The distribution of the corresponding state estimates is still consistent with the starting value.

### 4.2 Simulation analysis of data feature extraction based on iForest-LLE

To verify the accuracy and efficiency of iForest in extracting abnormal scores, the distribution, and variation of the Receiver Operating Characteristic (ROC) curve of iForest under different iTree numbers n and sampling numbers w are shown in Fig 5(A) and 5(B) below.

**Fig 5:** Distribution and changes of iForest ROC curve. (a) the different number n of iTree; (b) the different number w of samples.

As shown in the figure, when the corresponding number n of iTree is 10, iForest shows a relatively poor effect. When the corresponding number n of iTree is above 100, the detection effect of iForest is better. When the sampling number w corresponding to iTree is smaller than 10, the iForest algorithm model exhibits poor performance. When the sampling number w corresponding to iTree is greater than 10, the impact of the increase in the corresponding sampling number on the algorithm model is at a lower level. Therefore, the final determined number n of iTree in iForest is 100, and the number w of samples is 10.

The article "The data dimensionality reduction and bad data detection in the process of smart grid reconstruction through machine learning" was retracted in 2025. Reasons: unreliable results or conclusions; concerns about the results or conclusions; concerns about the peer review.

### 4.3 Verification of data attack detection model

To verify the performance of the attack detection model, the Ac distribution and changes in the detection model in the IEEE14-bus node system under different attack intensities are shown in Fig 6 below.

**Fig 6:** Ac distribution and changes in the detection model in the node system under different attack intensities.

As shown in the figure, in the IEEE14-bus node system, the Ac of the detection method proposed in this study eventually tends to 99%, and the corresponding convergence speed under different attack intensities is different. When the corresponding attack intensity (AI) is 0.1, the initial Ac value corresponding to the detection model is relatively low, which is around 92%, and the corresponding convergence speed is relatively slow. Ac increases with the increase in AI, and the corresponding convergence speed also becomes faster.

To further verify the effectiveness of the detection model proposed in this study, it is compared with other traditional detection methods. The AI is set to 1.0, and the distribution and changes of Ac in the IEEE14-bus node system are shown in Fig 7 below.

**Fig 7:** Comparison of Ac distribution and changes of several detection algorithms. DBN in the figure represents the deep confidence network algorithm.

As shown in the figure, the Ac value of each detection algorithm training phase is close to the test phase; at the same time, the Ac of each detection algorithm is distributed at above 90%. Furthermore, the performance of the detection algorithm model proposed in this study is superior to other traditional detection algorithms in terms of Ac and convergence speed. Its initial Ac is around 95%, and it eventually approaches 99%. This further validates the advantages of the proposed power data integrity detection algorithm model.

## 5. Discussion

The detection of FDIAs requires sufficient data samples as support. According to the actual situation, in this study, the data set is constructed based on the condition of incomplete network topology information. After the attack, the distribution of the state estimate value is consistent with the original distribution. Due to the attack, the value of the power measurement is changed, but as an entity, most of the state estimation residuals are consistent with the initial value. The state estimation residuals have not changed much compared with those before the attack. Therefore, in the IEEE14-bus node system and the IEEE118-bus node system, based on the incomplete network topology information conditions, it is still possible to achieve an injection attack against false data. Because of the high-dimensional and non-linear characteristics of power system data, comprehensively considering data dimensionality reduction and abnormal data processing, this study introduces the iForest algorithm and LLE construction to extract data features and realizes data dimensionality reduction operation and processing of abnormal score data. In the extraction of abnormal scores by the iForest algorithm, the learning scale of the algorithm is determined by the number corresponding to iTree. The analysis has found that the larger the number is, the better the improvement effect of the algorithm stability performance is, and the number of iTree samples can represent the size of the corresponding subspace of data samples. The fineness of iForest and iTree is determined by this parameter, and the analysis finds that the set value is not better when it gets larger. In the impact analysis of data feature extraction, the extraction of anomaly scores by the iForest algorithm has a greater impact on the realization of the data feature extraction effect.

The article "The data dimensionality reduction and bad data detection in the process of smart grid reconstruction through machine learning" was retracted in 2025. Reasons: unreliable results or conclusions; concerns about the results or conclusions; concerns about the peer review.

The traditional method for the detection of bad data in the power system can bypass the detection of bad data based on the residual error. By injecting false data into the measured values of the power system, an attack against the integrity of the power data can be achieved. However, the increase in the amount of data will lead to a reduction in detection accuracy and an increase in processing time. Considering the advantages of deep learning algorithms in the classification of massive data features, in addition to that the detection of FDIAs in power systems is a classification problem, the CNN-GRU hybrid network is introduced to construct the FDIAs detection model. The increase in AI led to the improvement of the accuracy of the model detection. CNN-GRU-based power data integrity attack detection shows good results, attacks targeting IEEE14-bus nodes system are easy to detect, and the performance and detection effect of the hybrid network-based algorithm detection model is superior to traditional detection methods, which expands the ideas of utilizing deep learning methods for the detection of bad data during the smart grid reconstruction process.

## 6. Conclusion

This study takes the detection of FDIAs as the starting point and selects the stable operation of the power system in the smart grid reconstruction as the research object. Through the establishment of attack datasets, feature data extraction methods based on isolated forests and locally linear embedding, and FDIAs detection models based on CNN, it is found that FDIAs can also be achieved under the condition of non-complete network topology information; the iForest algorithm has a greater influence in the extraction of anomaly scores; the introduction of machine learning and unsupervised dimensionality reduction methods have significantly improved the accuracy of FDIAs detection. However, the detection model proposed in this study is only suitable for attack detection under the condition of incomplete network topology information. In the future, the detection effect of other types of power data attack methods will be evaluated and the proposed method will be improved further.

The article "The data dimensionality reduction and bad data detection in the process of smart grid reconstruction through machine learning" was retracted in 2025. Reasons: unreliable results or conclusions; concerns about the results or conclusions; concerns about the peer review.

## Supporting information

S1 Data (XLSX)

## References

[1] ZhouZ, GaoC, ChenX, et al Social Big Data based Content Dissemination in Internet of Vehicles. IEEE Transactions on Industrial Informatics, 2018, 14(2), pp. 768–777.

[2] ZhangH, QiY, WuJ, et al DoS Attack Energy Management Against Remote State Estimation. IEEE Transactions on Control of Network Systems, 2018, 5(1), pp. 383–394.

[3] Tautz-WeinertJ, Watson SJ. Using SCADA data for wind turbine condition monitoring—A review. Iet Renewable Power Generation, 2017, 11(4), pp. 382–394.

[4] AshokA, GovindarasuM, AjjarapuV. Online Detection of Stealthy False Data Injection Attacks in Power System State Estimation. IEEE Transactions on Smart Grid, 2016, (99), pp. 1–1.

[5] Krsman VD, Sarić AT. Bad Area Detection and Whitening Transformation-based Identification in Three-Phase Distribution State Estimation. Iet Generation Transmission & Distribution, 2017, 11(9), pp. 2351–2361.

[6] SorrentinoE, AyalaC. Measurement of fault resistances in transmission lines by using recorded signals at both line ends. Electric Power Systems Research, 2016, 140, pp. 116–120.

[7] McMullen JG, McQuadeR, OgierJ, et al Variable virulence phenotype of Xenorhabdus bovienii (γ-Proteobacteria: Enterobacteriaceae) in the absence of their vector hosts. Microbiology, 2017, 163(4), pp. 510 10.1099/mic.0.000449 28430102PMC7008216

[8] ZhangJ, SankarL. Physical System Consequences of Unobservable State-and-Topology Cyber-Physical Attacks. IEEE Transactions on Smart Grid, 2016, 7(4), pp. 1–1.

[9] Herbst EB, UnnikrishnanS, WangS, et al The Use of Acoustic Radiation Force Decorrelation-Weighted Pulse Inversion for Enhanced Ultrasound Contrast Imaging. Investigative Radiology, 2016, 52(2), pp. 1.10.1097/RLI.0000000000000313PMC520925227495188

[10] LiX, LinY, XuY, et al Greedy Hybrid Beamforming for Multiuser MmWave MIMO Systems. Iet Communications, 2018, 11(18), pp. 2800–2805.

[11] Basart JP, ZhengY. Modeling very large array phase data by the Box-Jenkins method. Radio Science, 2016, 21(5), pp. 863–881.

The article "The data dimensionality reduction and bad data detection in the process of smart grid reconstruction through machine learning" was retracted in 2025. Reasons: unreliable results or conclusions; concerns about the results or conclusions; concerns about the peer review.

[12] MohammadpourfardM, SamiA, Seifi AR. A Statistical Unsupervised Method Against False Data Injection Attacks: A Visualization-Based Approach. Expert Systems with Applications, 2017, 84(oct.), pp. 242–261.

[13] Beg OA, Johnson TT, DavoudiA. Detection of False-Data Injection Attacks in Cyber-Physical DC Microgrids. IEEE Transactions on Industrial Informatics, 2017, 13(5), pp. 2693–2703.

[14] GanjkhaniM, Fallah SN, BadakhshanS, et al A Novel Detection Algorithm to Identify False Data Injection Attacks on Power System State Estimation. Energies, 2019, 12(11), pp. 2209.

[15] MoslemiR, MesbahiA, Mohammadpour VelniJ. Design of robust profitable false data injection attacks in multi-settlement electricity markets. Iet Generation Transmission & Distribution, 2018, 12(6), pp. 1263–1270.

[16] HosseinH, Taghi B SM. Designing three indicators to detect false data injection attacks on smart grid by dynamic state estimation. Journal of Intelligent and Fuzzy Systems, 2018, 35, pp. 1–12.

[17] WangQ, TaiW, TangY, et al A two-layer game theoretical attack-defense model for a false data injection attack against power systems. International Journal of Electrical Power & Energy Systems, 2019, 104(JAN.), pp. 169–177.

[18] CheL, LiuX, LiZ, et al False Data Injection Attacks Induced Sequential Outages in Power Systems. IEEE Transactions on Power Systems, 2019, 34(2), pp. 1513–1523.

[19] WangX, LuoX, ZhangM, et al Distributed detection and isolation of false data injection attacks in smart grids via nonlinear unknown input observers. International Journal of Electrical Power & Energy Systems, 2019, 110(SEP.), pp. 208–222.

[20] ShangF, WangB, YanF, et al Multidevice False Data Injection Attack Models of ADS-B Multilateration Systems. Security and Communication Networks, 2019, 2019, pp. 1–11.

[21] ZhangJ, ChuZ, SankarL, et al Can Attackers With Limited Information Exploit Historical Data to Mount Successful False Data Injection Attacks on Power Systems?. IEEE Transactions on Power Systems, 2018, 33(5), pp. 4775–4786.

[22] SreenathJ G, ChakrabartiS, RajawatK. Hierarchical Parallel Dynamic Estimator of States for Interconnected Power System. Iet Generation Transmission & Distribution, 2018, 12(10), pp. 2299–2306.

[23] SorrentinoE, AyalaC. Measurement of fault resistances in transmission lines by using recorded signals at both line ends. Electric Power Systems Research, 2016, 140, pp. 116–120.

[24] GonçalvesF M P, GoyderD J. A brief botanical survey into Kumbira forest, an isolated patch of Guineo-Congolian biome. Phytokeys, 2016, 65(65), pp. 1–14.10.3897/phytokeys.65.8679PMC495701827489484

The article "The data dimensionality reduction and bad data detection in the process of smart grid reconstruction through machine learning" was retracted in 2025. Reasons: unreliable results or conclusions; concerns about the results or conclusions; concerns about the peer review.

[25] ZhangS, MaZ, TanH. On the Equivalence of HLLE and LTSA. IEEE Transactions on Cybernetics, 2017, (99), pp. 1–12.10.1109/TCYB.2017.265533828166517

[26] Schneider WF, GuoH. Machine Learning. Journal of Physical Chemistry A, 2018, 122(4), pp. 879–879.10.1021/acs.jpca.8b0003429385808

[27] UmeharaK, OtaJ, IshidaT. Application of Super-Resolution Convolutional Neural Network for Enhancing Image Resolution in Chest CT. Journal of Digital Imaging, 2018, 31(4), pp. 441 10.1007/s10278-017-0033-z 29047035PMC6113156

[28] WangG M, QiaoJ F, BiJ, et al TL-GDBN: Growing Deep Belief Network With Transfer Learning. IEEE Transactions on Automation ence and Engineering, 2018, (2), pp. 1–12.

